The article "Cloning and Prokaryotic Expression of Carotenoid Cleavage Dioxygenases from Mulberry (Morus notabilis)" was published in 2022. Journal: Evid Based Complement Alternat Med.

# Cloning and Prokaryotic Expression of Carotenoid Cleavage Dioxygenases from Mulberry (*Morus notabilis*)

**DOI:** 10.1155/2022/4811144

**Published:** 2022-08-04

**Authors:** Dan Liu, Changyu Qiu, Xiaomei Lu, Yanrong Zeng, Chaohua Zhang, Tao Li, Guangshu Zhu, Ji He, Qiang Lin

**Affiliations:** Sericulture Technology Promotion Station of Guangxi Zhuang Autonomous Region, Nan Ning 530000, China

## Abstract

Carotenoid cleavage dioxygenase (CCD) is the key enzyme for carotenoid cleavage, and the products of carotenoid cleavage regulate the ability of plants to stress. In this paper, six *CCD* genes were obtained from *Morus notabilis* (Mn) by reverse transcription-polymerase chain reaction (RT-PCR) and we classified them into three subgroups based on gene structures and phylogenetic analysis. The CDS (coding sequence) regions of the six *MnCCD* genes were 1617, 1620, 1635, 1713, 1746, and 1791 bp in full length, encoding 538, 539, 544, 570, 581, and 596 amino acids, respectively. Then, Pcold–TF-*MnCCD* plasmids were constructed and independently transferred into *E. coli* BL21 (DE3), and the MnCCD proteins were successfully expressed by prokaryotic expression with an expected molecular weight of recombinant proteins (∼120 kDa) and high solubility. These results will lay a foundation for the identification of mulberry carotenoid products.

## 1. Introduction

A carotenoid is a kind of pigment widely distributed in nature [1, 2]. Its cleavage products are also precursors for the synthesis of a variety of active substances, which play an important role in plant stress response, growth, and development [3, 4]. Carotenoid cleavage oxygenase (CCO) is the key enzyme for carotenoid cleavage, including two subfamilies of CCD and 9-*cis epoxy* carotenoid dioxygenase (NCED) [5]. In *Arabidopsis*, the CCO family contains a total of nine genes, five of which belong to the NCED subfamily and are involved in the formation of abscisic acid precursors; the other four (AtCCD1, AtCCD4, AtCCD7, and AtCCD8) belong to the CCD subfamily and are involved in the cleavage of various carotenoids [6].

The products of carotenoid cleavage dioxygenase involve multiple biological processes including light sensation and hormone signaling and also contribute to the production of compounds related to smell and color [7, 8]. Moreover, this activity is of great significance in the process of the plant stress response. Studies have shown that carotenoid cleavage products (apocarotenoids) can improve the symbiosis efficiency of mycorrhizal fungi (AM), and AM can coexist with plant roots, thereby improving plant absorption of water and mineral nutrients, reducing plant absorption of heavy metal ions (copper, chromium, etc.), and ultimately helping plants resist stress [9–11]. In *Arbuscular mycorrhiza* of wheat, corn, and barley, carotenoids were cleaved into C_13_ and C_14_ apocarotenoids, and these apocarotenoids can also increase the *Mycorrhiza* symbiosis efficiency [12, 13]. So far, the *CCD* genes were subsequently isolated in a variety of plants, such as maize, tobacco, pepper, and saccharum [14–17]. Moreover, the carotene cleavage pathway in many species has been studied very clearly, for example, melon, tomato, osmanthus, and morning glory [18–21]. Specifically, the cleavage substrate and action site of CCD1 in different plants are not the same, but their products are involved in the production of flavors and aromas commonly [22, 23]. CCD2 is currently only found in the crocus plant, *Crocus sativus*, and CsCCD2 cleaves zeaxanthin and finally generates crocetin dialdehyde [8], so that the stigma of saffron appears yellow, orange, and red [24]. CCD4 has different cleavage sites in different plants. For example, the CCD4 of potatoes cleaved all-trans-*β*carotene to produce *β*-ionone (Market et al., 2015). Also, some plants such as CCD4 of citrus can cleave *β*-cryptoxanthin and zeaxanthin at the 7,8 (7′,8′) positions to synthesize *β*-orange pigment, whereas CCD7 and CCD8 are involved in the synthesis of strigolactone [25]. Even though extensive research has been performed on the function of *CCD* gene, little is known about the enzyme activity characteristics of CCD. The key to studying the characteristics of enzyme activity is to obtain the active CCD protein *in vivo*. Hence, this study aimed to successfully express the MnCCD proteins from the supernatant, that is, the soluble protein, which can lay a solid foundation for the subsequent enzymatic activity experiments. First, the cDNA of the six *MnCCD* genes were cloned from the young fresh leaves of mulberry by reverse transcriptase-polymerase chain reaction (RT-PCR). Furthermore, six MnCCD proteins were successfully obtained by prokaryotic expression.

The article "Cloning and Prokaryotic Expression of Carotenoid Cleavage Dioxygenases from Mulberry (Morus notabilis)" was published in 2022. Journal: Evid Based Complement Alternat Med.

## 2. Materials and Methods

### 2.1. Chemicals and Reagents

Phosphate-buffered solution (PBS) was obtained from Shanghai Biological Engineering Co. of China (Shanghai, China). The plant RNA extraction kit, reverse transcription kit, quantitative PCR kit, BCA protein assay kits, and His-tag Protein Purification Kit were purchased from Ruize Biological Technology Co. Ltd. (Nanning, China). Strains of *Escherichia coli* (*E. coli*) and Pcold–TF vector were kept in our laboratory.

### 2.2. Cloning of MnCCD Genes

*CCD* gene sequences from mulberry (Mn012507, Mn012508, Mn012509, Mn008739, Mn008741, Mn023189, GenBank ID: EXB32777.1, EXB32778.1, EXB32779.1, EXB58585.1, EXB58586.1, and EXC17835.1) were retrieved from the Mulberry Genome Database (https://morus.swu.edu.cn/morusdb/) and NCBI database (https://www.ncbi.nlm.nih.gov), and *CCD* genes in other plants (GenBank ID: NP_189064.1, NP_188062.1, NP_193569.1, NP_177960.1, etc.) were retrieved from the NCBI database. Multiple sequence alignment was performed with the ClustalX2.1 software. Quantitative PCR and full-length primers for six *MnCCD* genes were designed using Premier 5.0 (Table 1). Total RNAs were extracted from roots and leaves of mulberry using a plant RNA extraction kit according to the manufacturer's instructions. First-strand cDNA was produced using the reverse transcription kit and used as a template for PCR amplification. The amplification programme used for PCR is as follows: 95°C for 5 min, 32 cycles, 95°C for 30 s, 60°C for 30 s, 72°C for 90 s, and 72°C for 10 min. The products were separated on 1.0% agarose gels and cloned into the pMD19-T vector (TaKaRa, Dalian, China) to verify the sequence. The bioinformatic analysis tools were used with reference to the method of Liu et al. [26]. Putative N-terminal chloroplast transit and conservative domain predictions of MnCCDs were analyzed using the ProtParam tool (https://web.expasy.org/protparam/), ChloroP 1.1 Server (https://www.cbs.dtu.dk/services/ChloroP/), and conserved domains available online (https://www.ncbi.nlm.nih.gov/Structure/cdd/wrpsb.cgi). A schematic diagram of the gene structure of MnCCDs was drawn using the Exon–Intron Graphic Maker (https://www.wormweb.org/exonintron).

### 2.3. Expression and Purification of Recombinant MnCCD Proteins

The coding region of the six *MnCCD* genes containing the homologous sequence of Pcold–TF vector was cloned with the correct sequenced plasmid as a template. Then, the Pcold–TF vector and the target gene fragment were connected by homologous recombination. The correctly sequenced Pcold–TF-MnCCD plasmids were independently transferred into *E. coli* BL21 (DE3) and grown to OD about 0.6 for recombinant protein expression.The recombinant protein was expressed and purified with reference to the method of Liu et al. [26].

## 3. Results

### 3.1. Isolation of CCDs from *M. notabilis*

Six *CCD* genes were obtained in mulberry, and the six cloned *MnCCD* genes were *Mn008739*, *Mn008741*, *Mn012507*, *Mn012508*, *Mn012509*, and *Mn023189* and the open reading frames of the six genes were 1617, 1620, 1635, 1713, 1746, and 1791 bp (Figure 1), encoding proteins of 538, 539, 544, 570, 581, and 596 amino acids, respectively (Figure 2).

### 3.2. Bioinformatic Analysis of MnCCDs

The protein sequences of MnCCD proteins were compared and analyzed with reported CCD protein sequences from other species using ClustalX2.1 local software (Figure 2). Then, the related phylogenetic tree was obtained through the software MEGA5 (Figure 3). According to the evolutionary tree, plant carotenoid cleavage dioxygenases were divided into five subfamilies, CCD1, CCD2, CCD4, CCD7, and CCD8. The CCDs in plants were named according to the genetic relationship and homology of *Arabidopsis* CCDs (AtCCDs). From the phylogenetic tree, it can be seen that Mn012507, Mn012508, and Mn012509 are closely related to AtCCD1, so they were named MnCCD1A, MnCCD1B1, and MnCCD1B2, respectively. Mn023189 has the closest relationship with AtCCD4, so it was named MnCCD4. However, Mn008739, Mn008741, PaCCD1 (*Populus alba*), and JmCCD1 (*Juglans microcarpa*) are grouped together separately.

The article "Cloning and Prokaryotic Expression of Carotenoid Cleavage Dioxygenases from Mulberry (Morus notabilis)" was published in 2022. Journal: Evid Based Complement Alternat Med.

Mulberry CCD belongs to the RPE65 superfamily and the proteins of the MnCCD subfamily do not contain signal peptides or chloroplast transit peptides (except MnCCD4 and Mn008741), Notably, only MnCCD4 is localized in the chloroplast, the rest of the MnCCDs were localized in the cytoplasm, which may be related to their functional differentiation (Figure 4.).

### 3.3. Heterologous Expression and Purification of MnCCDs

There was a heavily expressed band at ∼50 kDa on SDS-PAGE in the control group and this is consistent with the predicted molecular weight of the tagged protein. However, the sample groups showed a heavily expressed new band at ∼120 kDa on SDS-PAGE and consistent with the expected molecular weight of the recombinant protein (Figure 5(a)). This result indicates the recombinant protein has been successfully expressed. Moreover, the six MnCCD crude protein samples were purified by nickel affinity chromatography and the eluted fractions were detected by SDS-PAGE electrophoresis and the positions of the purified six target proteins in 300 mM imidazole eluate were consistent with the predicted recombinant MnCCD proteins after Coomassie brilliant blue staining. Notably, there was only one obvious band in the sample group and the molecular weight was ∼120 kDa (Figure 5(b)). This shows that we have successfully purified the active target proteins from the supernatant.

## 4. Discussion

The number of *CCD* genes varies in different species. For example, 12, 11, and 10 *CCD* genes were identified in *Pyrus bretschneideri*, *Fragaria vesca*, and *Prunus persica*, respectively, and the phylogenetic tree clustered these genes into five branches CCD1, CCD4, CCD7, CCD8, and CCD-like [27]. Even in different varieties of the same species, the classification of *CCD* genes is different. In the case of sugarcane, *S. spontaneum* has 38 *CCD* genes and they were divided into seven groups, while the *CCD*s from R570 were 11 and were classified into five groups, missing CCD4 and CCD7in R570 compared to *S. spontaneum* [28]. In this study, the phylogenetic tree showed that the candidate *MnCCD*s clustered into three subfamilies: MnCCD1, MnCCD4, and CCD1-like (Mn008739 and Mn008741). Mn008739 and Mn008741 were clustered with PaCCD1 and JmCCD1, but they were independent of CCD1 of other plants, so Mn008739 and Mn008741 were named MnCCD1-like, as CCD7 and CCD8 were lost in *Morus notabilis,* this may be related to incomplete genomic information.

The article "Cloning and Prokaryotic Expression of Carotenoid Cleavage Dioxygenases from Mulberry (Morus notabilis)" was published in 2022. Journal: Evid Based Complement Alternat Med.

Eukaryotic and prokaryotic expression systems are commonly used to express recombinant proteins. Regardless of the expression system, the choice of vector and host cell is critical. Prokaryotic systems are more widely used because of their ability to obtain large quantities of recombinant proteins in a short period of time. The system is mainly based on *E. coli*, although *Bacillus* species are increasingly used [29]. Usually, different expression strains can be selected according to different needs. For example, Rosetta (DE3) PLySs is a highly stringent expression strain that can control expression levels and provide tRNAs with rare codons. Moreover, plasmid expression vectors include promoters, multiple cloning sites, terminators, replicons, signal peptides, fusion tags, and selectable markers. According to these characteristics of the vector, there are a variety of plasmids to choose from. Common prokaryotic expression vectors include pBAD, pET, POW3.0, and an expression vector for expressing GST fusion protein. Pet can express foreign proteins at a high level in host bacteria such as *E.coli* BL21 (DE3). Since the expressed proteins contain calmodulin-binding polypeptides and thrombin cleavage points, they are widely used in the purification industry. In this study, the pET32a vector was chosen as the expression vector, while the six recombinant MnCCD proteins did not express in the supernatant, it only expressed in a large amount in the precipitate, that is, it expressed in the form of inclusion bodies. Afterwards, we optimized the experimental conditions, and the situation remained the same. Finally, we reselected a vector, Pcold–TF, which provides cold-shock inducibility and triggers the expression of factors to improve the correct folding of the protein, thereby enabling soluble expression of recombinant proteins. Fortunately, we successfully expressed the six recombinant MnCCD proteins in the supernatant.

## 5. Conclusion

We identified six *CCD* genes from mulberry. Furthermore, we successfully obtained the MnCCD recombinant proteins by prokaryotic expression. The results showed that all MnCCD genes including CCD1-like genes could encode active carotenoid cleavage dioxygenases. These results lay the foundation for the analysis of the cleavage pathway of mulberry carotenoids.

The article "Cloning and Prokaryotic Expression of Carotenoid Cleavage Dioxygenases from Mulberry (Morus notabilis)" was published in 2022. Journal: Evid Based Complement Alternat Med.

## Figures and Tables

**Figure 1:** Multiple sequence alignment of six deduced MnCCD sequences. Conserved histidine residues are marked with a red asterisk.

**Figure 2:** PCR amplification of MnCCD gene. M: 5000 bp marker. (1) Mn023189, (2) Mn008741, (3) Mn012508, (4) Mn012509, (6) Mn008739, and (7) Mn012507.

**Figure 3:** Phylogenetic tree analysis of MnCCDs with the other species. Circle symbols of different colors represent the carotenoid cleavage dioxygenases (CCDs) of mulberry (MnCCDs), and the letter with the same color means the same subfamily. At, *Arabidopsis thaliana*; Ta, *Triticum aestivumLinn*; Cs, *Camellia sinensis*; Os, *Oryza sativa*; Mn, *Morus notabilis* Schneid.; Sb, *Sorghum bicolor*; Cs, *Cannabis sativa*; Pt, *Populus trichocarpa*; Pav, Prunus *avium*; Sl, *Solanum lycopersicum*; Pa, *Populus alba*; Jm, *Juglans microcarpa*; Zm, *Zea mays*; GenBank numbers: AtCCD1(), AtCCD4(), AtCCD7(), AtCCD8(), TaCCD4 (QEX50885.1), TaCCD1 (QEX50880.1), TaCCD7 (ASW22783.1), SlCCD1A (NP_001234542.1), SlCCD1B1 (NP_001233838.1), SlCCD1B2 (NP_001310512.1), CsCCD1 (AYK03324.1), CsCCD4 (AYK03325.1), SlCCD1A (NP_001234542.1), SlCCD1B1 (NP_001233838.1), SlCCD1B2 (NP_001310512.1), SbCCD1 (AGN03859.1), SbCCD4 (AGN03860.1), CcCCD4B (ABC26012.1), CcCCD4A (ABC26011.1), MdCCD4 (ABY47995.1), MdCCD7 (AUZ82805.1), OsCCD7 (XP_015637185.1), OsCCD1 (ABA99624.2), OsCCD8A (sp|Q93VD5.1), CsCCD1 (XP_030493365.1), PtCCD4 (XP_024457659.1), PavCCD1 (XP_021820758.1), PaCCD1 (XP_034890793.1), JmCCD1 (XP_041018063.1) Mn012507 (EXB32777.1), Mn012508(EXB32778.1), Mn012509 (EXB32779.1), Mn008739 (EXB58585.1), Mn008741 (EXB58586.1), Mn023189 (EXC17835.1).

**Figure 4:** Abridged general view of the MnCCD gene structure. Orange triangle: transcription start site; white rectangles: 5′UTR; green rectangles: chloroplast transit peptide; red rectangles: RPE65 domain; black broken lines: introns; white polygons: 3′UTR.

**Figure 5:** SDS-PAGE analysis of MnCCD proteins expressed in *E. coli* BL21 (DE3) cells and their purification. M: 180 kDa protein marker. (a) Lane 1: control, lanes 2–7: Mn008741, MnCCD1B1, MnCCD1A, MnCCD4, MnCCD1B2, and Mn008739; (b) lanes 1–6: the purified MnCCD proteins. Target protein bands are marked with black boxes, and the tagged protein band is marked with a red box.

**Table 1:** Primers used in this study.

Gene	Primer (5′-3′)	Used for
*MnCCD1A*	ATGGCGGAAGTGGCGTC	RT-PCR
	GATATTCAGTTTGAGTCCGAGTA	

*MnCCD1A*	atggagctcggtaccATGGCGGAAGTGGCGTC	Prokaryotic expression vector construction
	caggtcgacaagcttgaattcGATATTCAGTTTGAGTCCGAGTA	

*MnCCD1B1*	ATGGCCGAAATAGTGGATGTGAAT	RT-PCR
	TAGGACACCATTCCCAACATCAA	

*MnCCD1B1*	atggagctcggtaccATGGCCGAAATAGTGGATGTGAAT	Prokaryotic expression vector construction
	caggtcgacaagcttgaattcTAGGACACCATTCCCAACATCAA	

*MnCCD1B2*	GTGGGACTGTTCAAGGC	RT-PCR
	CTCTGCTGGGCAAATC	

*MnCCD1B2*	atggagctcggtaccATGGCGGAGAAGCCGAGC	Prokaryotic expression vector construction
	caggtcgacaagcttgaattcGAGTTTTGCTTGTTCTTGCAGTTG	

*MnCCD4*	ATGGCTTCCTCTTTTTTGGCAC	RT-PCR
	TCATGCCTGGTGAACCAAGTCC	

*MnCCD4*	atggagctcggtaccATGGCTTCCTCTTTTTTGGCAC	Prokaryotic expression vector construction
	caggtcgacaagcttgaattcTCATGCCTGGTGAACCAAGTCC	

*Mn008739*	ATGCCACATCACGTCTCCAA	RT-PCR
	CACCGAGACTGGTATGAAAGCT	

*Mn008739*	atggagctcggtaccATGCCACATCACGTCTCCAA	Prokaryotic expression vector construction
	caggtcgacaagcttgaattcCACCGAGACTGGTATGAAAGCT	

*Mn008741*	ATGGCATCATCGTATATGGCAT	RT-PCR
	TGGTGAGATTGGTATGAAAGCT	

*Mn008741*	atggagctcggtaccATGGCATCATCGTATATGGCAT	Prokaryotic expression vector construction
	caggtcgacaagcttgaattcTGGTGAGATTGGTATGAAAGCT	

Lowercase letters represent the homology arms containing *Kpn I* or *ECOR I* restriction sites.

The article "Cloning and Prokaryotic Expression of Carotenoid Cleavage Dioxygenases from Mulberry (Morus notabilis)" was published in 2022. Journal: Evid Based Complement Alternat Med.

## Data Availability

The data used to support the findings of this study are included within the article.
